# Strontium/Chitosan/Hydroxyapatite/Norcantharidin Composite That Inhibits Osteosarcoma and Promotes Osteogenesis In Vitro

This article has been retracted.

**DOI:** 10.1155/2020/9825073

**Published:** 2020-01-30

**Authors:** Zhipeng Huang, Haoyuan Sun, Yang Lu, Fengnian Zhao, Chang Liu, Qinglong Wang, Changming Zheng, Renpei Lu, Keguan Song

**Affiliations:** The First Affiliated Hospital of Harbin Medical University, No. 23 Post Street, Nangang District, Harbin, Heilongjiang, China

## Abstract

Hydroxyapatite can deliver drugs, and its composite material is capable of repairing bone defects in tumors. This study was conducted to evaluate the effect of composite materials on tumor growth inhibition and bone growth induction. Composites containing drug delivery compounds were synthesized by coprecipitation and freeze-drying and then characterized by scanning electron microscopy (SEM), X-ray diffraction (XRD), and Fourier-transform infrared spectroscopy (FTIR). In addition, the effect of hydroxyapatite nanoparticles (nano-SHAP) on proliferation of an osteosarcoma cell line (MG-63) and an osteoblast cell line (MC3T3-E1) was evaluated, and its mechanism was studied. The use of nano-SHAP alone did not affect the proliferation of normal cell lines. However, nanoparticles containing different amounts of norcantharidin in the composite materials and had different inhibitory effects on osteosarcoma and different effects on osteoblasts. And, with the increase of the content of norcantharidin, the antitumor performance of the composite has been enhanced. In summary, the nano-SHAP system developed in this study is a drug delivery material that can inhibit the growth of tumors and induce the proliferation of osteoblasts.

## 1. Introduction

Osteosarcoma (OS) is the most common primary malignant solid tumor in humans between the ages of 10 and 25 [1]. It is characterized mainly by the destruction of and recurrence in local tissue and is prone to distant metastasis. The widely accepted treatment for OS, which includes routine surgical resection and neoadjuvant chemotherapy, can improve the short-term survival rate to 60−70% [2]. However, tumor cells can remain in the area around the tumor resection site after surgery, resulting in high recurrence and bone destruction. Adjuvant chemotherapy plays an important role in killing the residual tumor cells and preventing tumor metastasis and recurrence [3]. In addition, it is common knowledge that bone defects need to be repaired using repair techniques such as allogeneic bone transplantation, iliac bone grafts, and irradiation bone grafts. However, there are still disadvantages in these technologies. For example, allogeneic bone is one of the most commonly used materials used for repairing tumor-induced bone defects, but it has no antitumor effect and is associated with the spread of infectious diseases and immune response [4]. Therefore, biocompatible biomaterials have the potential to be anticancer agents and to repair defects.

Composite materials, which comprise two or more excellent biomaterials, exhibit the properties of those materials. In recent years, composite materials composed of inorganic and organic components have attracted increasing attention. Depending on the characteristics of the components, the composites are used in catalysts, genes, and drug carriers [5, 6], for photodynamic and photothermal effects [7], and for their antibacterial properties [8, 9]. The organic components are important for modifying the inorganic materials, improving biocompatibility, escaping mononuclear cell phagocytic systems, and improving the therapeutic effects of the composite [10]. The cited studies have shown that composite materials will have a wide range of applications in the biomedical field and in many different scientific fields in the future.

Inorganic salts and carbohydrates play a crucial role in antitumor, bone regeneration, and biomineralization. Chitosan (CS) is the only basic aminopolysaccharide found in natural polysaccharides. It is widely used in many fields because of its biocompatible, biodegradable, and good antibacterial and antioxidant properties. CS can be used to absorb metal ions or other chemicals which is used to resist tumors [11]. Nanohydroxyapatite (nHAP) is the main inorganic component of human bones and teeth, accounting for 50–70% of human bone. Due to its good biocompatibility, biological activity, and osteoinductivity, nHAP added to the CS material can increase mechanical performance and mimic the natural structure of bone while maintaining biocompatibility [12]. In addition, studies have shown that CS/nHAP materials increase bone regeneration primarily by upregulating osteogenic genes and promoting mesenchymal stem cell (MSC) differentiation mineralization in vivo [13, 14]. Due to the advantages of good stability, biocompatibility, bone conductivity, and bone induction, CS/nHAP materials have been developed as osteogenic materials.

Strontium (Sr) ions not only promote the formation of new bone but also inhibit bone resorption [15], which have positive effects on promoting osteogenic differentiation of MSCs, preventing the proliferation of osteoclasts [16], and increasing the osteoinductivity of the composite. Marie et al. [17] reported that low-dose Sr^2+^ can accelerate bone formation and increase bone mass in animals. In the study by Lei et al. [15], SrHAP/CS was shown to have excellent cell compatibility and that it supports adhesion, diffusion, and proliferation of human bone marrow stromal cells (hBMSCs). Sr^2+^ released by the material contributed to osteogenic differentiation, and the presence of Sr in the SrHAP/CS material enhanced alkaline phosphatase (ALP) activity, extracellular matrix (ECM) mineralization, and the expression of osteogenesis-related genes Col-1 and ALP. Furthermore, the percentage of Sr in SrHAP had a large effect on ALP activity. ALP activity gradually increased as the Sr/Ca ratio in SrHAP increased and reached the maximum when the Sr/Ca ratio was 1 : 1. A high dose of Sr may lead to bone mineralization defects and even cause bone abnormalities.

Norcantharidin (NCTD) (7-oxabicyclo[2.2.1]heptane-2,3-dicarboxylic anhydride) is a new anticancer drug extracted and synthesized from traditional Chinese medicine. It has remarkable anti-cancer properties and is the only antitumor drug that can elevate white blood cell counts. Previous studies have demonstrated that NCTD suppresses the growth of numerous cancer cell lines, including oral cancer [18], hepatoma [19], and prostate cancer [20], via apoptosis, autophagy, and cell cycle arrest. Demethylcantharidin tablets have been used in the clinical treatment of hepatocellular, esophageal, and gastric cancer and leukemia [21]. It is reported that NCTD can play an anti-osteosarcoma role in many ways. NCTD can inhibit the proliferation of osteosarcoma cells by blocking the Akt/mTOR signal transduction pathway and inducing G2/M cell cycle arrest in 143B and SJSA osteosarcoma cells in a dose- and time-dependent manner. At the same time, NCTD led to the upregulation of cleaved caspase-3 and an increase in the downstream target cleaved PARP, which suggested that the extrinsic pathway may also be involved in NCTD-induced cell apoptosis [22]. By evaluating the effects of NCTD on OS cell lines (MG63 and HOS) in vitro and in vivo, we found that NCTD can inhibit cell cycle and induce apoptosis of human OS cells. These effects are mediated by autophagy induction, triggering ER stress and inactivation of the c-Met/Akt/mTOR pathway [23]. It works when the proliferation and apoptosis of normal cells are out of balance by inhibiting and then inducing apoptosis of tumor cells [24]. Studies have shown that 5 *μ*M of cantharidin kills nearly 45% of viable tumor cells [25]. In addition, 10 *μ*M of cantharidin was used to treat cells for different time periods and then western blot was used to analyze protein levels. Cantharidin increased the levels of p21 and phospho-p53 but decreased the levels of cyclin *E* and Cdc25c, which cause G0/G1 arrest [26]. NCTD effectively induces TNBC cell senescence and cell cycle arrest in vitro, accompanied by a decrease in phosphorylation of Akt and ERK1/2 and an increase in p21 and p16 [27]. At present, the most common route of administration is oral administration, which can lead to adverse reactions, such as nausea and vomiting. However, we have not found any reports that NCTD can be used as a composite biomaterial with anticancer effect in human body. However, to the best of our knowledge, few biomaterials can effectively kill residual tumor cells and repair bone defects after OS surgery. For the first time, we tried to incorporate NCTD into biological composite materials, which not only can reduce the systemic side effects caused by high blood drug concentration but also provide a good method and attempt for anti-osteosarcoma and osteogenesis.

In this study, we developed a novel strontium/chitosan/hydroxyapatite/norcantharidin (Sr/CS/HAP/NCTD or SCHN) composite that has certain osteoinductive properties and a significant inhibitory effect on the proliferation of OS cells. Experiments demonstrated that the inhibitory effect induced apoptosis by upregulating the expression of proapoptotic genes. In addition, the composite material reduced the osteoclastic activity of tumor cells by downregulating osteoclast-related genes. The composite shows good potential for treating OS in situ and repairing tumor-related bone defects.

## 2. Materials and Methods

### 2.1. Synthesis of Materials

SCHN composites were prepared by the method of in situ precipitation. The specific methods are as follows: three grams of CS powder (2% w/v; Sigma Aldrich, St. Louis, Mo, USA) was dissolved in 2% acetic acid solution and mechanical mixed at 60°C until the solution was clarified. SrCl_2_ 42 g and Ca(OH)_2_ 12 g were added into deionized water in proper sequence. After stirring and mixing smoothly, 30 g KH_2_PO_4_ was added slowly to keep the ratio of (Ca + Sr)/P at 1.67 and pH at 10, which was mixed for 24 hours. The above two solutions were mixed and divided into four parts, adding 0 g, 5/6 g, 5/3 g, and 5/2 g norcantharidin, respectively. The above liquids were fully mixed and added to 24-hole plate which was freeze-dried overnight in a freeze-dryer at −60°C. The mixtures were marked as Strontium/chitosan/hydroxyapatite/norcantharidin0, Strontium/chitosan/hydroxyapatite/norcantharidin1, Strontium/chitosan/hydroxyapatite/norcantharidin2, and Strontium/chitosan/hydroxyapatite/norcantharidin3. To facilitate the marking, we refer to above materials as Q0, Q1, Q2, and Q3.

### 2.2. Characterization of Materials

#### 2.2.1. Surface Microstructure

The surface microstructure and morphology of the samples were examined using a field-emission scanning electron microscope (FE-SEM, Quanta 200, Thermo Fisher Scientific, Waltham, MA, USA) at an acceleration voltage of 20 kV. All samples were plated with Au for 30 s before undergoing SEM. In addition, the microscope was equipped with an energy-dispersive X-ray (EDX) spectrometer to perform elemental analysis of the composite.

#### 2.2.2. Chemical Composition

The chemical composition of the composite was obtained using an FTIR spectrometer (Nicolet 6700, Thermo Fisher Scientific). The spectra of the Q0–Q3 materials were recorded using the KBr particle method with a 4000−400 cm^−1^ FTIR spectrophotometer. Each infrared spectrum was the average of 32 scans collected at 4 cm^−1^ resolution at 25°C over a range of 400−4000 cm^−1^.

#### 2.2.3. Elemental Analysis

The elemental analysis of the crystal phase exhibited on the powder was performed via X-ray diffraction (XRD) with a stepwise scanning diffractometer (XPS, Rigaku, Tokyo, Japan) equipped with Cu K*α* radiation target generated at 40 kV and 30 mA. The data set was collected in a 2*θ* range of 10°–70° at 0.02° per step.

#### 2.2.4. Swelling Behavior

The swelling behavior of the materials was evaluated using conventional methods [28]. Briefly, the dry weight of the material was recorded. Then, the material was immersed in 37°C phosphate-buffered saline (PBS), the wet weight was recorded for 1 hour and 24 hours, and the surface moisture was removed using filter paper. The expansion ratio was calculated using the following equation:

(1) $$\begin{array}{c} \text{Swell ratio}=\frac{\left(\text{Wet weight}-\text{dry weight}\right)}{\text{Dry weight}}. \end{array}$$

#### 2.2.5. Hemolysis Test

The method used had been reported previously [29]. Briefly, blood-containing EDTA was taken from volunteers and diluted to a blood : physiological saline ratio of 4 : 5. After 15 mg of the different composite materials was placed in 1 ml of normal saline, the mixture was incubated at 37°C for 30 min. Deionized water and PBS (each 1 ml) were added as positive and negative controls, respectively, followed by the addition of 200 *μ*l of diluted blood to each sample. The mixture was incubated in a constant temperature water bath at 37°C for 60 minutes. Finally, 100 *μ*l of the supernatant was transferred to a 96-well plate after centrifugation. The optical density (OD) was measured at 545 nm using a microplate reader.

### 2.3. Biological Properties of Materials

#### 2.3.1. Cell Proliferation and Toxicity

CCK-8 was used to measure the proliferation of osteogenic MC3T3-E1 cells and osteosarcoma MG-63 cells in the environment of composite immersion solution. In brief, 100 *μ*l of MC3T3-E1 cells or MG-63 cell suspension was seeded at a density of 2 × 10^4^ cells/ml in 96-well plates separately; culture medium and solution immersed in NCTD composites with different concentrations are added in proper order, which are cultured at 37°C. After 1, 4, and 7 days of incubation, the original culture solution was replaced by 10% CCK-8 culture solution in order to measure the OD value at 450 nm. The cell viability was calculated as follows:

(2) $$\begin{array}{c} \text{cell survival rate}=\left[\frac{A_{\text{s}}-A_{\text{b}}}{A_{\text{c}}-A_{\text{b}}}\right]\times 100\%, \end{array}$$

where *A*_s_ is the experimental well, *A*_c_ is the control well, and *A*_b_ is the blank well. All experiments were performed in triplicate.

#### 2.3.2. Apoptosis and Necrosis

The OS cell suspension (500 *μ*l) was seeded at a density of 2 × 10^5^ cells/ml for 2 days and detected using a CYTOMICS FC 500 MCL flow cytometer (Beckman Coulter, Brea, CA, USA). Briefly, after the extract of the composite material was added to the cells, the supernatant and adherent cells were collected and centrifuged at 1000 rpm for 5 min. The cell pellet was resuspended in 100 *μ*l of PBS and incubated with 10 *μ*l of Annexin V-FITC and 5 *μ*l of PI labeling solution for 20 min at 24°C–28°C in the dark. Finally, the cells were analyzed using flow cytometry, and the results were analyzed via Cytomics FC500 flow cytometry CXP analysis.

#### 2.3.3. Real-Time Polymerase Chain Reaction (RT-PCR)

Expression of apoptosis- and osteoblast-associated genes was assessed using RT-PCR. MG-63 cells and MC3T3-E1 cells, respectively, were cultured with the composite extract for 3 days. Total cellular RNA was isolated using TRIzol. The RNA was separated into an aqueous phase by the addition of chloroform. The colorless upper aqueous phase was then transferred to a new 1.5 ml tube to which isopropanol was added to precipitate the RNA. Finally, the RNA was washed with 75% ethanol and dissolved in enzyme-free water. RNA concentration was determined using a NanoDrop™ 2000 spectrophotometer (Thermo Fisher Scientific). RNA from each sample was reverse transcribed into complementary DNA (cDNA) using a PrimeScript™ RT reagent kit (Takara Bio Inc., Kusatsu, Japan) according to the manufacturer's instructions. Gene expression level of ALP, runt-associated transcription factor 2 (Runx2), osteocalcin (OCN), osteopontin (OPN), caspase-3 (CASP3), caspase-9 (CASP9), and matrix metallopeptidase 9 (MMP9) were evaluated by using iTap Universal SYBR® Green Spermix (BIO-RAD). The relative expression level of each target gene was then calculated using the 2^−ΔΔCT^ method. The relative mRNA expression level of each gene was normalized to that of GAPDH.

### 2.4. Statistical Analysis

All data were recorded as mean ± standard deviation. One-way analysis of variance (ANOVA) was performed using GraphPad Prism 6.0 (GraphPad Software, San Diego, CA, USA). *p* < 0.05 was considered as significant difference.

## 3. Results and Discussion

### 3.1. Composite Properties

In situ precipitation is a common method for preparing Sr/CS/HAP materials. In situ CS/HAP composites have better mechanical and biological properties than the physically prepared materials. The addition of Sr can enhance the cell adhesion [30] and the expression of osteogenesis-related genes [31] and promote osteoblast differentiation [15]. More importantly, the addition of Sr enhances the strength of the composites and improves the solubility of hydroxyapatite [32]. The various shapes of the HAP particles in the CS/HAP composite and the size of the composite depend on the processing conditions. Figures 1(a)−1(d) shows the morphology of the synthesized nanoparticles. The SEM images show that the materials were porous, that the pore size of the Q1, Q2, and Q3 composite materials was smaller than that of Q0, that the materials were made of small needle-like or plate-like crystals, and that the structure changed with the addition of NCTD. The materials had an irregular three-dimensional (3D) structure, and their pores were tightly connected to each other. The 3D environment may enhance cell-cell interaction and promote cell biological activity [33, 34]. Thus, the prepared material may be suitable for bone repair.  Figure 1(e) shows the energy-dispersive X-ray (EDX) spectrum of the Sr/HAP nanoparticles with the characteristic bands of Ca and Sr. The (Sr + Ca)/P ratio was about 1.66, which is similar to that of standard HAP. These minerals are key components of bone and tooth tissue.

### 3.2. Elemental Analysis of Q0, Q1, Q2, and Q3

In the XRD spectra of Q0, Q1, Q2, and Q3, a narrow and pointed peak was detected at *θ* values of 24.98°, 31.6°, 40.82°, and 56.38°, respectively (Figure 2), which shows that all the diffraction peaks correspond to the reflection of the composition of the material. As the concentration of NCTD increased, the diffraction spectrum lines narrowed and became sharper. The peak at 22.2° indicated an increase in crystallinity and a decrease in molecular size [35]. Meanwhile, traces of other impurities were not detected by this technique.

### 3.3. Chemical Composition

The functional groups contained in the composites were analyzed by FTIR.  Figure 3 shows the representative FTIR spectra of the synthesized Q0 and Q1, Q2, and Q3 nanoparticles. The characteristic peaks of CS appear at 1668 and 1431 cm^−1^, which correspond to the bands of amide-I and amide-II, and the vibrational band at 1024 cm^−1^ corresponds to *C* = *O* stretching [9]. For NCTD, the band at 860 cm^−1^ is attributed to the characteristic band of OH stretching, which is also the characteristic band of HAP [36]. Compared with Q0, the tensile vibration in Q1, Q2, and Q3 was enhanced, indicating that the addition of NCTD into the material was successful.

### 3.4. Swelling Behavior

The swelling behavior of the material was determined by immersing the composite materials in PBS solution.  Figure 4 shows that the swelling rates of the composites were different; however, the calculated differences were not significant. In addition, the swelling rates of the four materials did not change significantly during the incubation period, indicating that they were very stable. The difference in the swelling ratio among the materials, as seen in Figure 4, may be due to experimental errors in the materials.

### 3.5. Biocompatibility and Osteoinductivity

In this study, blood compatibility plays an important role in biological materials. Good biological materials should not cause red blood cells to rupture. In a blood compatibility test with a positive control (deionized water), a negative control (PBS), and the sample groups, the positive control caused hemolysis, with the released hemoglobin making the solution red (Figure 5(a)). After centrifugation, the red blood cells in the test tubes containing the material and the negative control were sedimented and the supernatant was clear. A small amount of the layer containing red blood cells was placed under a microscope, and no cell rupture was observed. It can be concluded that the material does not cause acute hemolysis. On the other hand, it is well known that CS and HAP possess excellent histocompatibility in bone repair. Although the addition of NCTD to materials has a good antitumor effect, it may also be toxic to normal osteoblasts. CCK-8 was used to detect the cytotoxicity of the composite to MC3T3-E1 cells. In all time intervals, Q1 and Q2 scaffolds showed little toxicity; accordingly, the OD value increased with the increase of incubation time, while the OD value of Q3 did not change significantly. In conclusion, the results indicate that the appropriate concentration of NCTD composite has good biocompatibility to bone tissue.

### 3.6. Antitumor and Increased Osteoblast Characteristics

To determine the optimal concentration of NCTD in the material, the cytotoxic effect of NCTD on osteosarcoma MG-63 cells and on MC3T3-E1 cells was determined using the standard CCK-8 assay.  Figure 6 summarizes the cell viability of MG-63 and MC3T3-E1 cells after 1, 3, and 7 days of cultured with different NCTD concentrations.  Figure 6(a) shows that, according to the CCK-8 assay, the osteoblast cells cultured in the three extract media cultured on day 1 had relatively similar absorbances as that of the control group (Q0) (*p* > 0.05). After day 1, the absorbance values of all groups increased, meaning that the number of live cells increased. On day 3, the OD value and number of live cells of the Q2 group increased (*p* < 0.01), and the number of live cells of the Q3 group increased (*p* < 0.05). On day 7, the OD value and number of live cells of the Q1 group increased (*p* < 0.01), and the number of live cells of the Q2 group increased (*p* < 0.05). At the same time, the absorbance values of the other composite material groups were not statistically significant (*p* > 0.05).  Figure 6(b) shows the results for the OS cells. The OD value and the number of live cells in the Q1, Q2, and Q3 composites gradually decreased compared with the values for Q0 as the culture period increased. The Q1, Q2, and Q3 composites had a significant inhibitory effect (*p* < 0.01). On day 7, Q3 inhibited tumor growth better than Q1 and Q2 (*p* < 0.05). The results showed that different NCTD levels affect cell viability differently. The higher the tumor cell inhibition, the better the viability of normal cells. Considering the effect of the composite extracts on the osteoblasts, the Q2 concentration of NCTD is best at promoting osteogenesis and inhibiting the proliferation of bone tumor cells.

To demonstrate our hypothesis, on day 2 of the culturing of OS cells with the different composite extracts, samples were collected by flow cytometry for apoptosis analysis using Annexin V-FITC and PI.  Figure 7(a) shows that the Sr/CS/HAP material (Q0) induced about 6.3% apoptosis and 5% necrosis, whereas the apoptosis and necrosis rates of the Q1, Q2, and Q3 materials were 5% and 6.8%, 4.2% and 6.5%, and 3.7% and 9.7%, respectively.  Figure 7(b) results display the apoptosis rate of Q2 and Q3 was significantly higher than that of Q0 (*p* < 0.05), Q2 was significantly higher than that of Q1 (*p* < 0.05), Q3 was significantly higher than that of Q1 (*p* < 0.01). The necrosis rate of Q1 was significantly higher than that of Q0 (*p* < 0.05), Q3 was significantly higher than that of Q0 (*p* < 0.001), and Q3 was significantly higher than that of Q1 and Q2 (*p* < 0.01), indicating that the addition of NCTD significantly induced apoptosis of the OS cells. Apoptosis increased with the increase in the concentration of NCTD, which is consistent with recent research [37].

In addition, osteolytic bone resorption is common in OS due to the osteolytic nature of OS cells. NCTD inhibits protein, DNA, and RNA syntheses, so we quantified the expression of OS, osteoblasts, and osteogenic-related genes in the different composites. Apoptosis regulation involves two major pathways: the mitochondria-mediated endogenous pathway and the caspase-dependent exogenous pathway [38]. In the caspase-dependent exogenous pathway, caspase-3 and caspase-9 are activated, which in turn leads to the cleavage of PARP [39]. Our study demonstrated that modification of the composite results in the upregulation of cleaved caspase-3, suggesting that the exogenous pathway may be involved in inducing apoptosis. Studies have shown that NCTD induces cell shrinkage, nuclear fragmentation, and chromatin condensation in OS cells, which possibly induce apoptosis through exogenous pathways [36]. MMP-9 degrades gelatin and collagen and is closely related to the bone destruction caused by OS invasion.  Figure 7(c) shows that the relative expression of CAS3 and CAS9 was higher in Q3 than in Q0 (*p* < 0.05) and that the expression of MMP9 in OS in the Q3 material was significantly lower than that in the Q0 composite (*p* < 0.05).

Figure 7(d) shows the mRNA expression levels of the osteogenic-related genes after osteoblasts were cultured in the composite extracts for 14 days. After 14 days of culture, the expression levels of Runx2, ALP, and OCN genes in the Q1, Q2, and Q3 composites were significantly higher than those in the control group, but the expression levels of the osteopontin (OPN) gene were significantly lower than that of the control group. In addition, Q3 had the greatest effect on the expression of the osteogenic-related genes Runx2, ALP, OCN, and OPN (*p* < 0.01). Bone formation consists of three main phases: proliferation, extracellular matrix maturation, and mineralization. Both ALP activity and collagen secretion increase with early osteogenic differentiation of osteoblasts [40], and Runx2 is the most important transcription factor for early osteoblast differentiation [41]. It has been reported that runx2 knockout mice have systemic osteogenic mineralization [42]. Runx2 also plays a role in the activation of genes involved in osteoblast differentiation, including ALP and OCN. OCN is a late marker of osteoblast differentiation, and its products indicate the onset of ECM deposition [43]. The relative expression levels of the above molecular indices were further confirmed by RT-PCR, confirming our understanding of the results in Figure 7(d). However, the expression of OPN was downregulated. Previous studies have demonstrated that OPN inhibits proliferation and differentiation of MC3T3-E1 cells [44]. Results of another study suggested that OPN has the ability to promote reuptake of osteoclasts as an effective stimulator of osteoclast absorption [45]. Our results appear to be consistent with those of these studies, suggesting that OPN, an inhibitor of osteoblast differentiation, is inhibited by Sr/CS/HAP. The difference in the results of the composites with respect to osteogenesis and osteogenesis-related gene expression may be due to the difference in the level of NCTD in the composites. However, potential mechanisms and signaling pathways require further research.

## 4. Conclusion

In the treatment of osteosarcoma, bone induction and inhibition of tumor cell growth are the key and difficult points. The results showed that the material of norcantharidin composite biomaterial had good biocompatibility, which do well in antitumor properties in vitro and promoted the mineralization of osteoblasts effectively. We believe that the strontium/chitosan/hydroxyapatite/norcantharidin composite biomaterials have a positive impact on the treatment of osteosarcoma. This study may provide information for the introduction of promising implants in surgical resection for OS hindlimb reconstruction.

## Figures and Tables

**Figure 1:** (a)−(d) SEM images of the materials of the Q0, Q1, Q2, and Q3 composite materials, respectively. (e) EDX spectra of the nanoparticles.

**Figure 2:** X-ray diffraction spectra.

**Figure 3:** FTIR diffraction spectra.

**Figure 4:** Expansion behavior of composites in PBS.

**Figure 5:** Composite hemolysis test. (a) None of the four materials caused hemolysis. (b) Supernatant of the area that underwent absorbance testing. Each value is the mean ± standard deviation of three determinations.

**Figure 6:** Effect of composites on the activity and cell viability of (a) murine osteoblast cell line MC3T3-E1 and (b) human osteosarcoma cell line MG-63 treated with the composite extracts for 1, 3, and 7 days. Cell viability was assayed using the CCK-8 method. Each experiment was repeated three times. ^*∗*^*p* < 0.05 compared with Q0.

**Figure 7:** (a) Cells were treated with different material extracts for 72 h and then stained with annexin V-FITC and PI and analyzed by flow cytometry. (b) Necrosis and apoptosis rates of MG-63 cells in the material. Compared with Q0, the apoptosis rates of Q1, Q2, and Q3 were significantly higher. (c) Relative expression of osteogenic-related genes after 14 days of culture. All pro-osteogenic genes in Q3 were significantly higher. (d) Relative expression of apoptosis-related genes after 3 days of culture. All the genes were significantly in Q3 (^*∗*^*p* < 0.05; ^*∗∗*^*p* < 0.01; ^*∗∗∗*^*p* < 0.001) compared with the levels in Q0.

## Data Availability

The data used to support the findings of this study are available from the corresponding author upon request.
